This article has been retracted.

# Endoplasmic reticulum Ca^2+^ release causes Rieske iron–sulfur protein-mediated mitochondrial ROS generation in pulmonary artery smooth muscle cells

**DOI:** 10.1042/BSR20192414

**Published:** 2019-12-04

**Authors:** Dapeng Dong, Qiongyu Hao, Ping Zhang, Tao Wang, Fei Han, Xiaodong Liang, Zhenghua Fei

**Affiliations:** 1 Department of Respiratory and Critical Care Medicine, The First Affiliated Hospital of Wenzhou Medical University, Wenzhou 325000, China; 2 Division of Cancer Research and Training, Department of Internal Medicine, Charles Drew University of Medicine and Science, Los Angeles, CA 90059, U.S.A.; 3 David Geffen UCLA School of Medicine and UCLA Jonsson Comprehensive Cancer Center, Los Angeles, CA 90095, U.S.A.; 4 Radiation and Medical Oncology Department, The 1st Affiliated Hospital of Wenzhou Medical University, Wenzhou 325000, China; 5 The Key Laboratory of Urinary Tract Tumors and Calculi, Department of Urology Surgery, The First Affiliated Hospital of Xiamen University, Xiamen 361003, China; 6 Division of Radiological Sciences, Washington University School of Medicine in Saint Louis, MO 63110, U.S.A.; 7 Department of Pathology, Tongji Hospital, Tongji University School of Medicine, Shanghai 200065, China; 8 Department of Pathology, Yancheng Hospital Affiliated Southeast University, Yancheng, Jiangsu 224000, China

**Keywords:** Intracellular calcium, mitochondrial ROS, Ryanodine receptor

## Abstract

Mitochondrial reactive oxygen species (ROS) cause Ca^2+^ release from the endoplasmic reticulum (ER) via ryanodine receptors (RyRs) in pulmonary artery smooth muscle cells (PASMCs), playing an essential role in hypoxic pulmonary vasoconstriction (HPV). Here we tested a novel hypothesis that hypoxia-induced RyR-mediated Ca^2+^ release may, in turn, promote mitochondrial ROS generation contributing to hypoxic cellular responses in PASMCs. Our data reveal that application of caffeine to elevate intracellular Ca^2+^ concentration ([Ca^2+^]_i_) by activating RyRs results in a significant increase in ROS production in cytosol and mitochondria of PASMCs. Norepinephrine to increase [Ca^2+^]_i_ due to the opening of inositol 1,4,5-triphosphate receptors (IP3Rs) produces similar effects. Exogenous Ca^2+^ significantly increases mitochondrial-derived ROS generation as well. Ru360 also inhibits the hypoxic ROS production. The RyR antagonist tetracaine or RyR2 gene knockout (KO) suppresses hypoxia-induced responses as well. Inhibition of mitochondrial Ca^2+^ uptake with Ru360 eliminates N- and Ca^2+^-induced responses. RISP KD abolishes the hypoxia-induced ROS production in mitochondria of PASMCs. Rieske iron–sulfur protein (RISP) gene knockdown (KD) blocks caffeine- or NE-induced ROS production. Taken together, these findings have further demonstrated that ER Ca^2+^ release causes mitochondrial Ca^2+^ uptake and RISP-mediated ROS production; this novel local ER/mitochondrion communication-elicited, Ca^2+^-mediated, RISP-dependent ROS production may play a significant role in hypoxic cellular responses in PASMCs.

## Introduction

Calcium ions (Ca^2+^) are one of the most crucial intracellular second messengers, involved in a plethora of cellular functions including cell survival and death, muscle contraction, regulation of metabolism, and gene expression [1]. Hypoxia causes strong vasoconstriction in pulmonary arteries, termed hypoxic pulmonary vasoconstriction (HPV) [1]. This unique response is an important adaptive mechanism for pulmonary ventilation/perfusion matching in the lungs, but may also become a crucial pathological factor for pulmonary hypertension [2,3]. HPV results from an increase in intracellular Ca^2+^ concentration [Ca^2+^]_i_), which is mediated by multiple ion channels in PASMCs. A series of studies have revealed that ryanodine receptors (RyRs), the Ca^2+^ release channels on the Endoplasmic reticulum (ER), are important for the hypoxic increase in [Ca^2+^]_i_ and contraction in PASMCs [4–6]. All three known subtypes of RyRs (RyR1, RyR2, and RyR3) are involved in hypoxic Ca^2+^ and contractile responses in PASMCs. However, RyR2 is the most valuable player [7–9]. The hypoxic increase in [Ca^2+^]_i_ in PASMCs has been thought to be attributed to the enhanced production of intracellular reactive oxygen species (ROS) due to their specific effects on ion channels [10–13]. Mitochondria-derived ROS levels are regulated by intracellular Ca^2+^ levels. Indeed, ROS increase when mitochondria are exposed to high [Ca^2+^] and [Na^+^] [14,15]. The specific communication between mitochondrial ROS and RyR2-mediated Ca^2+^ release serves as an essential mechanism for hypoxic cellular responses in PASMCs. Notably, mitochondria are a primary source of the hypoxic production of intracellular ROS, which increases the activity of protein kinase C and NADPH oxidase, leading to further ROS production, i.e. ROS-induced ROS production (RIRP) in PASMCs [4,16–19]. The hypoxia-induced mitochondrial ROS predominantly produce at the complex III, in which Rieske iron–sulfur protein (RISP) acts as a dispensable molecule [20–22]. Rieske proteins are iron–sulfur protein (ISP) components of cytochrome bc_1_ complexes and cytochrome b_6_f complexes and responsible for electron transfer in some biological systems [23]. It is a unique [2Fe-2S] cluster in that one of the two Fe atoms is coordinated by two histidine residues rather than two cysteine residues [24].

Considering all the aforementioned descriptions, together with the fact that Ca^2+^ signaling is central to mitochondrial functions, possibly including ROS generation, in cardiac myocytes [25], we have proposed an exciting hypothesis that the hypoxia-induced, RyR2-mediated increase in [Ca^2+^]_i_ may promote mitochondrial ROS production, which provides a positive feedback revenue for the hypoxic ROS production, thereby contributing to attendant Ca^2+^ and contractile responses in PASMCs. To test our novel hypothesis, we first sought to determine whether direct Ca^2+^ addition could increase ROS production in isolated mitochondria from PASMCs. RyR-mediated Ca^2+^ release plays an important role in cellular responses in PASMCs, thus, we next examined whether ROS production was augmented as well in isolated mitochondria from PASMCs following application of the classic RyR agonist caffeine to induce Ca^2+^ release from the ER. With the intention of defining a potential mechanism for the enhanced mitochondrial-derived ROS production in PASMCs, as a result of RyR-dependent Ca^2+^ release by caffeine, we planned to investigate the effect of pharmacological inhibition of mitochondrial Ca^2+^ uptake with Ru360 and genetic suppression of RISP in mitochondrial complex III using lentiviral RISP shRNAs. To extend these studies, we conducted a set of experiments to assess whether inhibition of mitochondrial Ca^2+^ uptake with Ru360 and prevention of RyR2-mediated Ca^2+^ release with its antagonist tetracaine and gene knockout were able to block the hypoxia-induced mitochondrial derived ROS production in PASMCs.

## Materials and methods

### Preparation of PAs and PASMCs

Resistance (third and smaller intralobar) PAs free of endothelium and connective tissues were dissected from male C57/B6 mice at 2 months old. PASMCs were isolated from the dissected PAs using the two-step enzymatic digestion method, in which the arteries were digested with papain and then collagenase in physiological saline solution (PSS). The harvested PASMCs were cultured in modified Dulbecco’s minimal essential medium (DMEM) for three passages and used in experiments.

PAs and PASMCs from smooth muscle-conditional RyR2 gene knockout (KO) mice on C57/B6 background were obtained as the same as described above. RyR2 KO mice were generated by crossbreeding RyR2flox/flox mice with smooth muscle-specific myosin heavy chain Cre recombinase mice. The KO mice were genotyped by polymerase chain reaction analysis of tail tip DNAs. Western blot analysis revealed that these mice showed the absence of RyR2 expression in PAs.

### Detection of ROS production

ROS production in PASMCs was measured using chloromethyldihydrodichlorofluorescein diacetate (CM-H2DCF/DA) assay by ROS Detection Cell-Based Assay Kit (Item# 601520, CAYMAN CHEMICAL) according to the manufacturer’s protocol. Briefly, PASMCs were seeded in a black tissue culture treated 96-well plate at a desired concentration. Pyocyanin and N-acetyl Cysteine were designated as positive and negative control, respectively. Culture media were aspirated off and 150 µl of Cell-Based Assay Buffer were added in the well. Cell-Based Assay Buffer were aspirated off and a small amount of liquid were left in the well. About 130 µl of ROS Staining Buffer were added in each well. About 10 µl of N-acetyl Cysteine were added as negative control. Cell were covered and incubated at 37°C, protected from light. About 10 µl of Pyocyanin Working Reagent were added after 30-min incubation as positive control, and incubated for an additional hour at 37°C, protected from light. Staining buffer were aspirated carefully and 100 µl of Cell-Based Assay Buffer was added in the well. The assay plate were placed in the GloMax®-Multi Detection System (Promega), and the fluorescence was measured using an excitation wavelength between 480 and 500 nm and an emission wavelength between 510 and 550 nm. Mitochondrial ROS was measured using Mitochondrial ROS Detection Assay Kit (Item# 701600, CAYMAN CHEMICAL), according to the manufacturer’s protocol. Different concentrations of buffered Ca^2+^ or hypoxia were apply to respiration buffer and ROS was detected at 37°C using the GloMax®-Multi Detection System. Cytosolic ROS was also assessed using specific ROS biosensor pHyPer-cyto [26]. Primary cultured PASMCs were transfected with pHyPer-cyto construct. After transfection for 72 h, caffeine or norepinephrine was added to induce ROS production. HyPer was alternatively excited at 420 and 500 nm. Emitted fluorescence at 510 nm was measured at 37°C using the GloMax®-Multi Detection System.

Lucigenin and Redox Sensor Red CC-1 (Red CC-1) also detected ROS production in PASMCs and mitochondria. Lucigenin (20 μM, Molecular Probes, R-6868) was added to one well of 96-well plate which containing 1.5 × 10^5^ PASMCs or 10 μg mitochondria sample or 3 μg of complex III protein. Emitted chemiluminescence derived by lucigenin was detected by GloMax®-Multi Detection System. The initial (maximal) values of lucigenin-derived chemiluminescence were normalized to control group. As described previously [27,28], same amount of PASMCs and mitochondria samples as used in lucigenin assay were loaded at 37°C for 30 min with Red CC-1 (1 mM, Molecular Probes, R-14060). Red CC-1 derived fluorescence was measured using a GloMax®-Multi Detection System with an excitation wavelength of 544 nm and emission wavelength of 612 nm. Intracellular ROS production was determined by the difference in fluorescence between the wells containing the assay buffer with and without cells. Fluorescent intensity was normalized to control group.

### Intracellular calcium ([Ca^2+^]_i_) detection

Intracellular calcium were measured using Calcium Quantification Kit - Red Fluorescence (abcam, cat#: ab112115), according to the manufacturer’s protocol. Briefly, prepare a calcium standard by diluting the appropriate amount of the 300 mM Calcium Standard into H_2_O to produce a calcium concentration ranging from 0 to 3 mM (12 mg/dl). Add 50 μl of serial diluted calcium standard into each well. Add 50 μl of assay reaction mixture to each well of calcium standard, blank control, and test samples to make the total calcium assay volume of 100 μl/well. Incubate the reaction for 5–30 min at room temperature, protected from light. Monitor the fluorescence intensity with a fluorescence plate reader at *E*_x_/*E*_m_ = 540/590 nm.

### Intra-mitochondria calcium ([Ca^2+^]_mito_) detection with mutant aequorin

Mitochondria targeted calcium sensor pcDNA3.1+/mit-2mutAEQ (Asp119 to Ala, Asn28 to Leu points mutations on aequorin) was a gift from Javier Alvarez-Martin (Addgene plasmid # 45539). According to previous report, pcDNA3.1+/mit-2mutAEQ was purified and transfected to primary cultured mouse PASMCs. After transfection, PASMCs were incubated for 2 h at room temperature in standard medium [145 mM NaCl, 5 mM KCl, 1 mM MgCl_2_, 1 mM CaCl_2_, 10 mM glucose and 10 mM Hepes (pH 7.4)] with 2 μM coelenterazine w (Cat#10110-1, Biotium). After incubation, PASMCs were treated with different concentrations of caffeine and norepinephrine for 5 min. Luminescence intensities were recorded by luminometer. Luminescence unit was calibrated into Ca^2+^ concentration by following previous publications [29].

### RISP KD

Lentiviral shRNAs specific for RISP were used to knockdown its expression in PASMCs. Lentiviruses containing RISP shRNAs and non-silence shRNAs were purchased from ThermoScientific OpenBiosystems and then packaged using pCMV-dR8.2 dvpr and pCMV-VSV-G packing vectors. The efficiency of RISP KD was determined using Western blot analysis.

### Hypoxia

To induce hypoxic responses, samples were treated with a normoxic medium that was aerated with a 21% O_2_, 5% CO_2_ and 74% N_2_ mixture for 10 min and then hypoxic medium gassed with a 1% O_2_, 5% CO_2_ and 94% N_2_ mixture for 5 min. As a control, samples were treated with normoxic medium alone.

### Animal and ethics information

All animal experiments were performed at animal facility of Wenzhou Medical University according to an approved protocol by the Animal Care and Ethics Committee of Wenzhou Medical University. Male C57BL/6 mice bred under specific pathogen-free conditions were 8–10 weeks old at exposure initiation. All the investigations complied with the National Institutes of Health Guide for the Care and Use of Laboratory Animals.

### Statistical analysis

Levels of statistical significance were evaluated with data from no less than three independent experiments using one- or two-way ANOVA with an appropriate post hoc test. The differences between the means of data at *P* < 0.05 were considered statistically significant.

## Results

### Application of caffeine and norepinephrine to elevate [Ca^2+^]_i_ significantly increase ROS production in PASMCs

Caffeine triggers Ca^2+^ release by reducing the threshold for luminal Ca^2+^ activation of RyR2 [30]. Here, we first examined whether RyR-mediated Ca^2+^ release might cause ROS generation in PASMCs. Cells were treated with the classic RyR agonist caffeine (200 μM) for 5 min, ROS generation was remarkably increased in caffeine-treated cells compared with untreated cells by measuring DCFDA-derived fluorescence intensity (Figure 1A). Norepinephrine, a major vascular neurotransmitter, can increase [Ca^2+^]_i_ by largely inducing Ca^2+^ release from the ER via inositol 1,4,5-trisphosphate receptors (IP_3_Rs) in vascular SMCs [31]. Accordingly, we sought to test whether treatment with norepinephrine could also increase ROS production in PASMCs. Similar to caffeine, application of norepinephrine (20 μM) for 5 min resulted in an increase in intracellular ROS production in PASMCs (Figure 1A). Representative microscope images of DCFDA fluorescence were shown in Supplementary Figure S1A. We also observed that exposure of caffeine or norepinephrine facilitated Ca^2+^ release in cytosol (Figure 1B). Caffeine- and norepinephrine-induced ROS generation was also detected by Red CC-1-derived fluorescence intensity and lucigenin emitted chemiluminescence (Figure 1C,D). Similar to DCFDA method, these results confirmed that caffeine and norepinephrine could elicit intracellular ROS generation. Simultaneously, we found marked increase in Fluo-3 AM fluorescence of the cytosolic calcium levels after caffeine or NE treatment as compared with control in PASMCs (Figure 1G). Hypoxia or deoxygenated blood causes lower pressure and less vessel resistance in pulmonary arteries. However, in systemic arteries, i.e. mesentery arteries, transmitting deoxygenated blood leads to vessel constriction and increasing of vessel pressure. We speculate ER Ca^2+^ release induced ROS generation may show distinct functional difference between pulmonary arteries and mesentery arteries. As shown in Figure 1E, caffeine and norepinephrine were not able to induce ROS generation in cytosol of primary cultured mesentery artery smooth muscle cells (MASMCs); however, they elevated intracellular Ca^2+^ concentration (Figure 1F). ROS measurement in MASMCs were also performed by Red CC-1 and lucigenin (Supplementary Figures S2 and S3).

**Figure 1:** Elevation of [Ca^2+^]i by caffeine or norepinephrine increases ROS production in cytosol of PASMCs, but not MASMCs (**A**) PASMCs were treated with caffeine (200 μM) or norepinephrine (20 μM) for 5 min. Intracellular ROS generation was measured using DCFDA assay. (**B**) PASMCs were exposed to caffeine (200 μM) or norepinephrine (20 μM) for 5 min, and Ca^2+^ levels were then detected using a Ca^2+^ quantification kit. (**C**) Red CC-1 and lucigenin (**D**) assay was used to determine ROS generation in PASMCs. (**E**) MASMCs were treated with caffeine (200 μM) or norepinephrine (20 μM) for 5 min. Intracellular ROS generation was measured using DCFDA assay. (**F**) MASMCs were exposed to caffeine (200 μM) or norepinephrine (20 μM) for 5 min, and Ca^2+^ levels were then detected using a Ca^2+^ quantification kit. Data represent mean ± SEM; *n* = 6, *P < 0.05; **P < 0.01; ***P < 0.001, compared with control by two-tails Student’s *t* test. (**G**) Fluo3-AM staining of cytosolic Ca^2+^ ions in PASMCs. PASMCs were treated with caffeine (200 μM) or norepinephrine (20 μM) for 5 min, then stained with 0.5 μ M Fluo-3-AM in HBSS buffer.

### Inhibition of mitochondrial Ca^2+^ uptake blocks caffeine-induced ROS production in PASMCs and Ca^2+^-evoked ROS generation in mitochondria of PASMCs

It is known that mitochondria is central sources for intracellular ROS generation in PASMCs [32,33]. To further prove the role of Ca^2+^ in mitochondrial ROS production, we investigated the effect of caffeine, norepinephrine and hypoxia-induced increase in intramitochondria Ca^2+^ concentration [Ca^2+^]_mito_). Mitochondria targeted Ca^2+^ sensor pcDNA3.1+/mit-2mutAEQ generated luminescence intensity was calibrated with different concentration of buffered Ca^2+^ (Supplementary Figure S4). Norepinephrine and caffeine were exposed to pcDNA3.1+/mit-2mutAEQ transfected PASMCs. Emitted luminescence intensities were calibrated to [Ca^2+^]_mito_ concentration and quantified as dose–response curve. As shown in Figure 2A,B, caffeine and norepinephrine can increase [Ca^2+^]_mito_ in a dose-dependent manner. We assumed that caffeine- or NE-induced Ca^2+^ release might cause mitochondrial Ca^2+^ uptake, and accordingly mediate Ca^2+^-dependent mitochondrial ROS generation. To test this assumption, PASMCs were treated with Ru360 (1 µM), which is a mitochondria calcium uniporter (MCU) inhibitor [34], for 5 min, then exposed to caffeine (200 µM) or NE (20 µM) for 5 min in the presence of Ru360. As shown in Figure 2C,D, treatment with Ru360 attenuated caffeine- or NE-elicited ROS production in mitochondria. Previous study indicated that cell stimulation caused local hotspot of Ca^2+^ transients (20–40 μM), while the Ca^2+^ transients increase of the rest of cells is much less (1–2 μM) [35]. Activation of calcium-ion (Ca^2+^) channels on the plasma membrane and on intracellular Ca^2+^ stores, such as the endoplasmic reticulum, generates local transient increases in the cytosolic Ca^2+^ concentration that induce Ca^2+^ uptake by neighboring mitochondria. In order to clarify the effects of Ca^2+^ on mitochondria ROS generation, we designed different concentration of buffered Ca^2+^ to mimic local Ca^2+^ transient. Freshly isolated mitochondria from PASMCs were incubated with different concentrations of buffered Ca^2+^. As shown in Figure 2E, 1, 10 and 100 µM Ca^2+^ significantly changed mitochondrial ROS generation detected by DCFDA. In agreement with its effect on caffeine- or NE- induced responses, treatment with Ru360 blocked Ca^2+^-evoked ROS generation in isolated mitochondria (Figure 2E).

**Figure 2:** Caffeine or norepinephrine elevates mitochondrial ROS by mitochondrial Ca^2+^ influx ([Ca^2+^]_mito_) (**A**) [Ca^2+^]_mito_ was determined by mitochondria-targeted double-mutated aequorin (pcDNA3.1+/mit-2mutAEQ), which was described in ‘Materials and Methods’ section. Mitochondria Ca^2+^ uniporter inhibitor Ru360 (1 μM) decreased [Ca^2+^]_mito_ caused by caffeine or norepinephrine (**B** and** C**); PASMCs were treated with caffeine (200 μM) or norepinephrine (20 μM) (**D**) for 5 min. Mitochondrial ROS generation was measured using a Mitochondrial ROS Detection Assay Kit. (**E**) Freshly isolated mitochondria from PASMCs were exposed with different concentrations of Ca^2+^ in the presence or absence of Ru360 (1 μM); mitochondria ROS were determined by DCFDA assay. Data were obtained from three separate experiments. *P < 0.05; **P < 0.01; ***P < 0.001 compared with Ca^2+^ (0 μM) group.^ #^*P*<0.05, ^##^*P* < 0.01 compared Ca^2+^ (100 μM) with absence of Ru360 group.

### Inhibition of RyRs attenuates hypoxic ROS production in PASMCs

RyR-mediated Ca^2+^ release is essential for the hypoxic increase in [Ca^2+^]_i_ in PASMC [36,37]. Previous studies have shown that RyR1, RyR2 and RyR3 all are expressed and mediate acute hypoxic [Ca^2+^]_i_ and contractile responses in PASMCs; however, the role of RyR2 dominates over that of RyR1 and RyR3 [38,39]. To explore the role of RyRs in the hypoxic ROS generation in PASMCs, we treated PASMCs with the RyR antagonist tetracaine (1 µM) for 5 min and then exposed to hypoxia for 5 min. ROS generation was largely suppressed in PASMCs by treatment with tetracaine under hypoxic conditions (Figure 3A). We also examined the effect of RyR2 KO on the hypoxic ROS production in PASMCs. RyR2 KO PASMCs was isolated from RyR2 KO mice. Figure 3C showed no RyR2 protein expression in RyR2 KO PASMCs. As shown in (Figure 3D), acute hypoxic exposure caused ROS increase in PASMCs, but not in RyR2 KO PASMCs. Ca^2+^ release in cytosol by hypoxia treatment were also observed (Figure 3B,E). RyR2 KO also blocked NE induced mitochondrial ROS increase in PASMCs (Figure 3F).

**Figure 3:** Inhibition or genetic deletion of RyR2 blocks hypoxic ROS production in PASMCs (**A**) Intracellular ROS production was detected by DCFDA assay in PASMCs treated with RyRs inhibitor tetracaine (1 μM) for 5 min followed by hypoxia for 5 min. (**B**) Intracellular Ca^2+^ levels were then detected using a Ca^2+^ quantification kit. Data were obtained from three separate experiments. *P < 0.05; **P < 0.01; ***P < 0.001 compared with normoxic control group, and ^#^*P* < 0.05; ^##^*P* < 0.01 compared with hypoxic control group. (**C**) Western blots of RyR2 expression in WT and RyR2 KO PASMCs. (**D**) PASMCs from wild-type (WT) and RyR2 KO mice were exposed to normoxia or hypoxia for 5 min. ROS were measured in cells by DCFDA assay. (**E**) Intracellular Ca^2+^ levels were then detected using a Ca^2+^ quantification kit. Data were obtained from three separate experiments. **P < 0.01 compared with normoxic WT group, and ^##^*P* < 0.01 compared with hypoxic WT group. (**F**) Mitochondrial ROS generation upon NE treatment in WT and RyR2 KO PASMCs.

### Inhibition of RyRs and mitochondrial Ca^2+^ uptake block hypoxia-induced mitochondrial ROS production in PASMCs

We next determined ROS production in mitochondria of PASMCs following hypoxia exposure. We assessed the effect of RyRs on mitochondrial ROS production. The results indicated that mitochondrial ROS generation was increased by hypoxia treatment (Figure 4A). Inhibition of RyRs with tetracaine or IP3R with 2-APB attenuated hypoxia-induced ROS generation in mitochondria (Figure 4A,C). The hypoxic ROS increase was significantly suppressed in mitochondria from RyR2 KO PASMCs (Figure 4B). To evaluate mitochondrial ROS generation upon cytosolic [Ca^2+^]_i_ increase, PASMCs were treated with Ru360 for 5 min, then hypoxia was introduced for 5 min. As shown in Figure 4D, Ru360 abolished hypoxia-induced ROS generation in mitochondria. The elevation of [Ca^2+^]_mito_ was significantly inhibited by Ru360 (Figure 4E). RyR2 overexpression rescued mitochondrial ROS increase in RyR2 KO PASMCs (Figure 4F).

**Figure 4:** Inhibition or genetic deletion of RyR2 blocks hypoxic ROS production in mitochondria of PASMCs (**A**) PASMCs were pretreated with tetracaine (1 μM) (C) for 5 min followed by hypoxia for 5 min. Mitochondrial ROS generation was measured using a Mitochondrial ROS Detection Assay Kit. **P < 0.01 compared with normoxia control group, and ^##^*P* < 0.01 compared with hypoxia control group. (**B**) PASMCs from WT and RyR2 KO mice were exposed to normoxia or hypoxia for 5 min. Mitochondrial ROS were measured by a Mitochondrial ROS Detection Assay Kit. Data were obtained from three separate experiments. **P < 0.01 compared with control, and ^#^*P* < 0.05; ^##^*P* < 0.01 compared with WT group. (**C**) WT and RyR2 KO PASMCs were pretreated with 2-APB (20 μM) for 5 min followed by hypoxia. Mitochondrial ROS generation were measured using a Mitochondrial ROS Detection Assay Kit. **P < 0.01 compared with normoxia control group, and ^##^*P* < 0.01 compared with hypoxia control group group. (**D**) Cells were treated with Ru360 (1 μM) for 5 min, then exposed to caffeine (20 mM) for 5 min. mitochondrial ROS were measured by using a Mitochondrial ROS Detection Assay Kit. **P < 0.01; ***P < 0.001 compared with normoxia control group, and ^##^*P* < 0.01 compared with hypoxia control group. [Ca^2+^]_mito_ was determined by mitochondria-targeted double-mutated aequorin (pcDNA3.1+/mit-2mutAEQ). Ru360 (1 μM) decreased hypoxia-caused [Ca^2+^]_mito_. (**E**) RyR2 KO PASMCs were transfected with RyR2 overexpression plasmids. All groups were treated with hypoxia for 5 min. Mitochondrial ROS generation were measured using a Mitochondrial ROS Detection Assay Kit. **P < 0.01 compared with WT group, and ^#^*P* < 0.05 compared with WT RyR2 KO group.

### Rieske iron–sulfur protein gene silencing inhibits caffeine and hypoxia-induced ROS production in PASMCs and Ca^2+^-evoked ROS generation in mitochondria from PASMCs

Studies have shown that RISP is indispensable for the hypoxic ROS generation in PASMCs [40]. To determine the role of RISP in Ca^2+^-induced ROS generation, RISP shRNA was retrovirally transduced into PASMCs, data showed RISP protein expression were largely suppressed compared with non-infected or NS shRNA (Figure 5A). We also demonstrated that hypoxia-induced mitochondrial ROS generation was significantly inhibited in RISP-deficient PASMCs (Figure 5B). Moreover, knockdown RISP also slightly suppressed cytosolic hypoxia-ROS generation (Figure 5C). RISP overexpression rescued mitochondrial ROS increase in RISP KO PASMCs (Figure 5D). Caffeine-or NE-evoked mitochondrial ROS production was abolished in PASMCs infected with lentiviral RISP shRNAs (Figure 5E,G). However, Ca^2+^-induced ROS production in cytosol was slightly attenuated by RISP knockdown (Figure 5F,H).

**Figure 5:** RISP gene knockdown blocks hypoxia-, caffeine- or NE- induced ROS production in PASMCs (**A**) Western blots of RISP expression in PASMCs uninfected, infected with lentiviral RISP shRNA, and non-silencing (NS) shRNA. (**B**) Mitochondrial and Cytosolic ROS (**C**) were determined after hypoxia treatment. RISP knockdown inhibited hypoxia-induced ROS increase. Data were obtained from three separate experiments. **P < 0.01 compared with normoxia NS_shRNA group, and ^#^*P* < 0.05; ^##^*P* < 0.01 compared with hypoxia NS_shRNA groups. (**D**) RISP KO PASMCs were transfected with RISP overexpression plasmids. All groups were treated with hypoxia for 5 min. Mitochondrial ROS generation were measured using a Mitochondrial ROS Detection Assay Kit. **P < 0.01 compared with WT group, and ^#^*P* < 0.05 compared with WT RISP KO group. (**E**) PASMCs were treated with caffeine (200 μM) (**E** and**F**) or NE (20 μM) (**G** and** H**) for 5 min in non-infected, infected with non-silencing (NS) shRNA PASMCs or lentiviral encoding RISP shRNA. Mitochondria and Cytosolic ROS were determined after treatment. Data were obtained from three separate experiments. ***P < 0.001 compared with non-infected control group, and ^#^*P* < 0.05; ^##^*P* < 0.01 compared with caffeine-treated NS_shRNA group.

## Discussion

ROS-mediated increase in [Ca^2+^]_i_ plays an important role in hypoxia-induced pulmonary vasoconstriction, vasoremodeling and even hypertension [41,42]. Presumably, the talk of Ca^2+^ signaling to ROS signaling may enhance the hypoxia-induced ROS production in PASMCs, which provides a positive mechanism to mediate the hypoxic ROS production and associated cellular responses.

In the present study, we have also found that application of norepinephrine, a major neurotransmitter in vascular SMCs, to active α-adrenergic receptors and increased [Ca^2+^]_i_ can result in an increase in ROS generation as well in PASMCs. It is well known that activation of α-adrenergic receptors induces ER Ca^2+^ release by opening inositol 1,4.5-triphosphate receptors (IP3Rs). Ca^2+^ release via IP3Rs may activate adjacent RyRs to induce further ER Ca^2+^ release, i.e., a local Ca^2+^-induced Ca^2+^ release (CICR) process, in PASMCs [43,44]. Thus, the role of norepinephrine in inducing ROS production is likely to be, at least in part, implemented by RyR-dependent Ca^2+^ release as a result of local IP3R/RyR interaction-mediated CICR. Another novel finding is that the application of caffeine to activate RyRs on the ER and then to induce Ca^2+^ release by the ER can also cause a significant increase ROS production in isolated PASMCs. Mitochondria are a major source for ROS production in PASMCs, and mitochondrial ROS is primarily generated at complex III [45–48]. Consistent with these previous reports, the present study has also shown that Ca^2+^ release following activation of RyRs with caffeine increases ROS production in mitochondria from PASMCs. Application of norepinephrine, similar to caffeine, also results in an increase in ROS production as well in mitochondria from PASMCs. Moreover, by using mitochondria targeted Ca^2+^ sensor, we successfully measured and quantified the amount of Ca^2+^ changes inside the mitochondria induced by different concentrations of caffeine or norepinephrine. In complement of caffeine- and norepinephrine-induced responses, different concentrations of exogenous Ca^2+^ also significantly increase ROS production in isolated mitochondria from PASMCs. These data not only reveal that Ca^2+^ release from the ER may cause intracellular ROS production primarily at mitochondrial in PASMCs, but also further support our novel concept that the ER can locally communicate with closely neighboring mitochondria in a format of Ca^2+^-mediated ROS production in PASMCs.

We have surmised that the increased [Ca^2+^]_i_ may give rise to an increase in mitochondrial Ca^2+^ uptake, leading to ROS production in mitochondria. Consistent with our conjecture, treatment with Ru360, a specific mitochondrial Ca^2+^ uptake inhibitor [49], prevents caffeine from inducing ROS production in PASMCs. Likewise, Ru360 also blocks caffeine-induced ROS generation in mitochondria from PASMCs. More interestingly, Ru360 inhibits hypoxia-induced mitochondrial ROS production. These results reveal that mitochondrial Ca^2+^ uptake serves as a critical step for Ca^2+^-dependent ROS production, thereby playing an important role in hypoxic cellular responses in PASMCs.

Previous study have demonstrated that RyRs play an important role in hypoxia-induced increase in [Ca^2+^]_i_ in PASMCs and pulmonary vasoconstriction in PAs [50–53]. Hypoxia may inhibit voltage-dependent K^+^ (Kv) channels and activate store-operated Ca^2+^ (SOC) channels, leading to Ca^2+^ and contractile responses in PASMCs; however, the hypoxic inhibition of Kv channels and activation of SOC channels may be secondary to ER Ca^2+^ release, presumably via RyRs [51]. These data reinforce the importance of RyRs in hypoxic cellular responses in PASMCs. As such, we have assumed that hypoxia-induced, ROS-initiated, RyR-mediated ER Ca^2+^ release may cause further ROS production in PASMCs. Indeed, in the present study we have observed that treatment with tetracaine to block RyRs remarkably inhibits the hypoxic ROS production in PASMCs. Tetracaine also reduces the hypoxic response in isolated mitochondria from PASMCs. All three known RyR subtypes are involved in hypoxic Ca^2+^ and contractile responses in PASMCs; however, RyR2 is the most valuable player. In agreement with this notion, we have unveiled that hypoxia causes a much smaller increase in ROS production in PASMCs from RyR2 KO mice than control (WT) mice. Furthermore, the hypoxic ROS generation is significantly reduced in mitochondria from RyR2 KO mice. These pharmacological and genetic findings demonstrate that RyR2 functions as a key molecule to implement the focal communication from the ER to mitochondria, leading to Ca^2+^-dependent ROS production in PASMCs during hypoxic stimulation.

In support, Waypa et al. have also found that RISP gene depletion abolishes hypoxia-induced increase in [Ca^2+^]_i_ in pulmonary arteries and right ventricular systolic pressure [22]. In line with the importance role of RISP, in the present study we have discovered that RISP knockdown inhibits Ca^2+^- and caffeine-induced ROS production in mitochondria from PASMCs. We have also shown that RIPS plays an important role in hypoxia-induced increase in [Ca^2+^]_i_ in PASMCs. However, further experiments are needed to determine whether Ca^2+^ may produce a direct or an indirect effect on RISP-mediated mitochondrial ROS production in PASMCs.

Mitochondrial ROS are generated in both physiological and pathological conditions. On the one hand, moderate levels of ROS are involved in cell signaling by affecting the redox state of signaling proteins, Under physiological conditions, the balance between ROS generation and ROS scavenging is highly controlled [54]. However, on the other hand, excessive mROS are among the major determinants of toxicity in cells and organisms [55]. Physiological ROS levels initiate a wide array of cellular responses, ranging from triggering signaling pathways, activation of mitochondrial fission and autophagy, adaptation to hypoxic condition, and differentiation to regulation of aging-related processes [56]. In specific conditions, ROS production is induced in response to a stress and it functions as an intermediate signaling to facilitate cellular adaptation [57]. Thus, the study of the crosstalk between calcium and ROS in pathophysiological conditions might be useful to identify novel therapeutic strategies to cure pathologies characterized by dysregulation of mitochondrial Ca2+ homeostasis. In summary, the present study is the first time to demonstrate that Ca^2+^ release from the ER via RyRs or IP3Rs can increase [Ca^2+^]_i_, mitochondrial Ca^2+^ uptake, and RISP-dependent mitochondrial ROS production (Figure 6). This novel focal communication from the ER to mitochondria in the form of Ca^2+^-induced ROS production may play an important role in the overall hypoxia-induced mitochondrial RISP-dependent ROS production, thereby contributing to Ca^2+^ and contractile responses in PASMC.

**Figure 6:** ROS and Calcium crosstalk between endoplasmic reticulum and mitochondria The ER is a major site of calcium ions (Ca^2+^) storage within muscle cells. Calcium from ER cisternae is flowing mainly through calcium release channels as inositol 1,4,5-trisphosphate receptors (IP3R) and ryanodine receptors (RyR). High levels of calcium stimulate respiratory chain activity leading to higher amounts of reactive oxygen species (ROS) through RISP. ROS can further target ER-based calcium channels leading to increased release of calcium and further increased ROS levels.

## Highlights

- Agonist-induced ER Ca^2+^ release increases ROS production in mitochondria of PASMCs.
- Exogenous Ca^2+^ causes ROS production in isolated mitochondria. RYR2 antagonist or *Ryr2* KO, mitochondrial Ca^2+^ uptake inhibitor, RISP KD all prevent the hypoxic ROS production.
- ER/mitochondrion communication-elicited, Ca^2+^-mediated, RISP-dependent ROS production may significantly contribute to hypoxic cellular responses in PASMCs.

## Supplementary Material

Supplementary Figures S1-S5

## Abbreviations

[Ca^2+^]_i_: intracellular Ca^2+^ concentration
[Ca^2+^]_m_: mitochondrial Ca^2+^ concentration
ER: endoplasmic reticulum
HPV: hypoxic pulmonary vasoconstriction
IP3R: Inositol 1,4,5-trisphosphate Receptor
KD: knockdown
KO: knockout
PASMC: pulmonary artery smooth muscle cell
PSS: physiological saline solution
RIRP: ROS-induced ROS production
RISP: Rieske iron–sulfur protein
ROS: reactive oxygen species
RyR: Ryanodine Receptor
